# Different Characteristics and Interleukin-6 Ratios of Scattering-Type Aortic Plaques

**DOI:** 10.7759/cureus.52949

**Published:** 2024-01-25

**Authors:** Sei Komatsu, Chikao Yutani, Satoru Takahashi, Tomoki Ohara, Nobuzo Iwa, Mitsuhiko Takewa, Hirotaka Noda, Kazuhisa Kodama

**Affiliations:** 1 Department of Cardiology, Osaka Gyoumeikan Hospital, Osaka, JPN; 2 Department of Pathology, Osaka Gyoumeikan Hospital, Osaka, JPN; 3 Department of Medical Technology, Morinomiya University of Medical Sciences, Osaka, JPN

**Keywords:** interleukin-6, nonobstructive general angioscopy, cholesterol crystals, spontaneously ruptured aortic plaque, aorta

## Abstract

Background

Cholesterol crystals (CCs) are related to innate inflammation in spontaneously ruptured aortic plaques (SRAPs), and variability exists in the CCs and interleukin (IL)-6 ratio in SRAPs.

Methods

The prevalence of scattering-type ruptures that glittered against the light of angioscopic fibers (puff-chandelier ruptures) and those that did not (puff ruptures) was analyzed in 848 patients with suspected coronary artery disease. Overall, 177 puff-chandelier ruptures and 105 puff ruptures were sampled using nonobstructive general angioscopy (NOGA). The sampled plaques were analyzed by direct detection of CCs with polarized light microscopy. The characteristics of the plaque fragments from puff and puff-chandelier ruptures were compared. The Interleukin-6 (IL-6) ratios were calculated for 100 puff-chandelier ruptures and 100 puff ruptures.

Results

CCs were detected in 54% of puff-chandelier ruptures and 20% of puff ruptures. The longer and shorter dimensions of the puff ruptures were smaller than those of the puff-chandelier ruptures. CCs were more prevalent in puff chandeliers than in puff ruptures (54% vs. 20%, respectively; p<0.0001). The number of CCs was higher in puff chandeliers than in puff ruptures with CCs (median 12,727 (interquartile range (IQR) 3,636-25,909)/10 mL vs. median 3,182 ( IQR 909-9,318)/10 mL) in CC-positive samples (p=0.0120). The IL-6 ratio of puff-chandelier ruptures was higher than that of puff ruptures (p=0.0014).

Conclusions

Examination of plaque fragments from puff-chandelier and puff ruptures revealed a higher prevalence of CCs in puff-chandelier ruptures compared to puff ruptures. Puff chandeliers exhibited a significantly greater number of CCs, suggesting a potential correlation with inflammatory levels. The IL-6 ratio was also higher in puff-chandelier ruptures. Direct detection of CCs and hematoxylin and eosin staining for SRAPs demonstrated variations in CC degree and dimensions between puff-chandelier and puff ruptures. Puff-chandelier ruptures exhibited more CCs associated with innate inflammation and larger fragments than puff ruptures. NOGA proved effective in detecting diverse characteristics and inflammation levels, as indicated by IL-6, in scattering-type SRAPs.

## Introduction

Embolism by aortic plaques cause acute and chronic organ damage [1-4]. Using nonobstructive general angioscopy (NOGA), spontaneously ruptured aortic plaques (SRAPs) were observed in 80.9% of the patients with or suspected to have coronary heart disease [3,5]. The number of aortic plaques detected using NOGA is associated with cardiovascular events [6]. The frequency and number of SRAPs are associated with ischemic stroke [7]. There are two kinds of scattering-type SRAPs [4,8,9]. The first is a puff-chandelier rupture, where puff-like materials glow against the light from the NOGA fiber catheter tip and spontaneously blow out [3,5]. Using a new analysis method, cholesterol crystals (CCs) were found to be present in the puff-chandelier ruptures, and the crystals in the plaque were reflected against light in NOGA [3,9].

Embolism-induced end-organ damage may occur due to mechanical ischemia and inflammatory responses. CCs induce immune inflammation [10-12]. Recently, we reported a moderate correlation between CC count and the interleukin-6 (IL-6) ratio, that is, the IL-6 level in SRAPs was compared to that at the beginning of the aorta in situ [13]. Thus, CCs are related to innate inflammation in SRAPs, and variability exists in the CCs and IL-6 ratio in SRAPs. Plaque components, including CCs and inflammatory cytokines scattered by SRAPs, may cause inflammation at the embolization site.

The other scattering-type SRAP is a puff rupture, which can also blow out spontaneously but does not glisten against the angioscopic fiber light [5,8]. Thus, puff rupture is expected to include fewer CCs and have lower inflammatory levels than puff-chandelier rupture. NOGA can assess the characteristics of scattering-type ruptures, including inflammatory levels, if puff-chandelier ruptures and puff ruptures are distinguished by inflammatory levels. Assessing the inflammatory levels in SRAPs allows for precisely evaluating the effects of drugs such as anti-inflammatory agents [14-16]. This study aimed to compare the CC content characteristics and inflammatory levels between puff-chandelier ruptures and puff rupture SRAPs.

## Materials and methods

Patient recruitment

To assess the occurrence of puff-chandelier and puff ruptures, we included 848 consecutive patients with confirmed or suspected coronary artery disease. These individuals underwent both coronary angiography and aortic angioscopy for screening aortic atherosclerosis. The data for this analysis were drawn from the angioscopic database and encompassed the period from January 1, 2018, to December 31, 2022.

To identify the characteristics of scattering-type aortic ruptures, we evaluated 282 scattering-type plaques from the patients who underwent emergency or elective cardiac catheterization with scanning and sampling of SRAPs using NOGA at Osaka Gyoumeikan Hospital (University Hospital Medical Information Network Center ID: UMIN000047477). The exclusion criteria were as follows: patients with hemodynamic instability (i.e., Killip >2 or shock), rupture of aortic dissection, hypersensitivity to contrast agents, or under hemodialysis. This investigation was carried out following the principles outlined in the Declaration of Helsinki and was approved by the Ethics Committee of the Social Welfare Service Corporation, Osaka Gyoumeikan Hospital (approval number: 21-001). Written informed consent was obtained from all enrolled patients.

Angioscopic system

NOGA was performed using a 6-French (F) soft-chipped Ikari left 3.5 guiding catheter that could flexibly move in the aorta after coronary angiography or coronary intervention. The systems utilized in NOGA were VISIBLE Fiber (FT-203F, FiberTech Co. Ltd., Tokyo, Japan), an imaging system, and a console (Intertec Medicals Co. Ltd., Osaka, Japan). Scanning angioscopy of the aorta and the recording of images and videos were performed as previously described [3,5].

Prevalence of puff-chandelier and puff ruptures

NOGA scans the ascending aorta to the iliac artery to detect SRAPs [3-5]. SRAPs were defined as previously reported [8]. The prevalence of puff-chandelier and puff ruptures among the SRAPs was calculated. Puff ruptures were defined as materials that were scattered spontaneously like puffs, whereas puff-chandelier ruptures were defined as a mixture of the features of both puff rupture and chandelier appearance [5,8,9]. The numbers of puff-chandelier ruptures and puff ruptures were counted, and the median values were calculated.

Sample size calculation

We calculated a sample size of at least 100 in each group of scattering-type plaques based on the prevalence and the number. In a preliminary study, the prevalence of puff-chandelier rupture and puff rupture was found to be 70% and 80%, respectively. The ratio of the number of puff-chandelier ruptures and puff ruptures was 2:1. Plaques were randomly selected from the sampling database.

Sampling of SRAPs

The SRAP samples were obtained as previously described [4,9,16]. Briefly, puff-chandelier rupture and puff rupture were targeted for sampling. Blood was sampled from the 6-F guiding catheter. Blood (10 mL) was collected from each SRAP. Half of the samples were used to measure both high-sensitivity C-reactive protein (hs-CRP) and IL-6 levels, and the other half was used to measure the CC content. After sampling, the fiber catheter and the probing catheter were reinserted into the guiding catheter. Blood samples were applied to a filter paper [16].

Histological examination

Puff-chandelier SRAP samples on the filters were directly placed in 15% buffered formalin, decalcified, and embedded in paraffin for representative histological examinations. Sections (3-5 μm) including the tissues were stained with hematoxylin and eosin (H&E). Samples were also stained with an anti-human cluster of differentiation (CD)-68 for macrophages, anti-IL-1β, and anti-IL-6, as previously reported [9].

Counting visible debris

Generally, debris is visibly picked up by a needle on 150-200-μm filters in the aspiration catheter system. However, materials that appear as debris cannot be collected because they disappear on drying. Visible debris was defined as materials that well-trained doctors or technicians could pick up on filter paper. The number of visible pieces of debris was counted to determine the percentage yield rate of the general sampling method. Visible debris has approximately >300 μm of longer dimensions.

Detection of CCs and fibrin

The sampled plaques were analyzed using CC direct detection without solvents and conventional H&E staining [3,9,17]. During the H&E staining preparation, CCs were dissolved in solvents such as ethanol and xylene. Two methods were used for the direct detection of CCs; if either method detected CCs, they were considered present.

Direct Detection of CCs: Quantitative and Qualitative Analyses of CCs

Direct CC detection is divided into quantitative and qualitative analyses [3,17]. For quantitative analyses, 22 µL of blood from each sample was placed between a powderless glass slide and a glass cover [16]. The glass was affixed to the resin along the edges of the glass cover and exposed to ultraviolet rays for 30 minutes to avoid drying. Sampled blood with the glasses was instantly frozen to -20 °C and then thawed gently to a room temperature of 25 °C for erythrocyte hemolysis (instant freeze and thaw method) [17]. The count of multilayer and monolayer CCs was conducted through polarized light microscopy by a pathologist with expertise in reviewing a minimum of 1,000 samples in this domain. The determination of the number of multilayer CCs involved adjusting the focus for each CC layer. The expression of the CC count per 22 µL was standardized to 10 mL, corresponding to the sampled blood volume of 10 mL.

The sampled blood was subjected to a qualitative analysis of CCs by rinsing the filter paper with distilled water and identifying the CCs in the resulting solution. A more precise method was reported by Iwa et al. [17]. A positive result for CCs was obtained if either quantitative or qualitative analysis detected CCs. Polarized light microscopy was used to detect the CCs in the blood placed on the filters, and the solution content was obtained after rinsing the filter. The samples were tested in a blinded manner.

Conventional Histological Examination

Histological examination was performed if filter paper or visible debris on the filters was found in the sampled SRAPs. The identified materials were directly immersed in 15% buffered formalin for decalcification. Subsequently, the specimens were embedded in paraffin, and transverse sections of the tissues, measuring 3-5 mm in thickness, were stained with H&E for standard histological analysis.

Measuring the dimensions of plaques

The long and short sides of the plaques in the H&E-stained sections were measured for 100 randomly selected samples, as previously reported [3] using ImageJ software version 1.53a (National Institutes of Health, Bethesda, Maryland, United States).

Analysis of IL-6 level and IL-6 ratio

Serum IL-6 levels were measured with a commercially available assay reported previously [13]. We defined the IL-6 ratio as the ratio of the serum IL-6 level in SRAPs to the IL-6 level at the beginning of the aorta, that at the sinus of Valsalva was defined as the baseline value. The IL-6 ratio was calculated in 100 randomly selected puff-chandelier ruptures and 100 puff ruptures in the same manner [13]. The IL-6 levels and ratios between puff-chandelier and puff ruptures were compared.

Analyzing the correlation between serum IL-6 levels and hs-CRP levels

IL-6 and hs-CRP levels in the peripheral arteries were measured. Regression analysis was performed to analyze the correlation between serum IL-6 and hs-CRP levels in the 100 samples. IL-6 and hs-CRP levels in SRAPs were measured as previously described. Regression analysis was performed to analyze the correlation between IL-6 and hs-CRP levels in the SRAPs of the 50 samples.

Statistical analyses

Statistical analyses were conducted with the JMP statistical software (version 16.0.1; SAS Institute, North Carolina, United States). The number of CCs and lengths of the long and short sides of the plaques were expressed as medians (interquartile range (IQR)). The incidence of visible debris, the percentage of valid samples for H&E staining, the detection rate of CCs, the ratio of atheroma diagnoses, the ratio of fibrin diagnoses, and the ratio of undeterminable samples were compared using the Chi-square test. The number of CCs and the long and short sides of the plaques in puff and puff-chandelier ruptures were compared using analysis of variance. IL-6 levels and IL-6 ratios of the sampled materials in the puff-chandelier and puff ruptures were compared using analysis of variance. Two-tailed p-values <0.05 were considered statistically significant.

## Results

Analyzed plaques were 177 puff-chandelier ruptures and 105 puff ruptures from 157 patients (102 males and 55 females). Patient characteristics are presented in Table 1, and representative images, schemas, and videos of the puff-chandelier and puff ruptures are shown in Figure 1 and Video 1.

**Table 1:** Patients’ characteristics

Characteristics	Occurrence group (N=848)	Sampling group (N=157)
Gender (Male), n (%)	548 (65%)	101 (64%)
Age (years), mean ± SD	72 ± 10	72 ± 11
Hypertension, n (%)	601 (73%)	107 (68%)
Diabetes, n (%)	298 (36%)	63 (40%)
HbA1c (%), mean ± SD	6.1± 3.4	6.0± 1.1
Fasting blood glucose (mg/dL), mean ± SD	121± 52	121± 50
Dyslipidemia, n (%)	495 (67%)	91 (58%)
Triglyceride (mg/dL), mean ± SD	138± 92	155± 104
High-density lipoprotein cholesterol (mg/dL), mean ± SD	52± 15	50± 15
Low-density lipoprotein cholesterol (mg/dL), mean ± SD	95± 38	104± 38
C-reactive protein (mg/dL), mean ± SD	0.73± 5.46	0.51± 1.16
History of cerebral infarction, n (%)	-	19 (12%)
History of low extremity artery disease, n (%)	-	19 (12%)

**Figure 1:** Representative images and schemas of two kinds of scattering-type ruptures detected by nonobstructive angioscopy. (A) Puff-chandelier rupture; (B) Puff rupture

**Video 1:** Representative video of puff-chandelier rupture and puff rupture

Among the 848 patients, puff-chandelier ruptures and puff ruptures were detected in 559 (66%) and 633 (75%) patients, respectively. The median numbers of puff-chandelier and puff ruptures per patient were 2 (IQR, 0-5) and 1 (IQR, 0-4), respectively. Representative histological and immunohistological images of the SRAPs are shown in Figure 2.

**Figure 2:** Representative histological and immunohistological images of the spontaneously ruptured aortic plaques. (A) Histopathological images of SRAPs (bar, 20 μm): Representative images of hematoxylin and eosin-stained sections. The needle-shaped empty clefts have been regarded as CCs; (B–D) Immunostaining of debris from SRAPs (bar, 20 μm); (B) Image of immunostaining for CD68, revealing the presence of M. Vacant clefts, that were traces of CCs, are surrounded by M. Representative images of immunostaining for IL-1β (C) and IL-6; (D) IL-1β and IL-6 staining of macrophages IL-1β, Interleukin-1β; IL-6, Interleukin-6; M, macrophages; SRAP, spontaneously ruptured aortic plaque; CC, cholesterol crystal

Detection of CCs and dimensions of plaques in puff-chandelier ruptures

A total of 177 puff-chandelier ruptures were sampled. Visible debris was detected in 46 samples (26%) and CCs were directly detected in 95 samples (54%) using polarized light microscopy (Figure 3). In total, 135 samples (76%) contained materials that could be diagnosed by H&E staining of filter papers fixed in formalin, and 42 samples (24%) did not contain any plaque material. Fifty-one samples were analyzed as atheromas, and fibrin was detected in 84 samples using H&E staining. All 51 samples contained empty needle-shaped clefts, suggesting dissolved CCs. The median values of the long and short sides of the plaques were 76 μm(IQR 49-122μm) and 41 (IQR 24-83μm), respectively. 

**Figure 3:** Flow chart of the detection of cholesterol crystals using direct detection and hematoxylin and eosin staining from 177 puff-chandelier ruptures.

Detection of CCs and dimensions of plaques in puff ruptures

A total of 105 puff ruptures were sampled, and visible debris was detected in 14 samples (13%) (Figure 4). CCs were directly detected in 21 samples (20%) by polarized light microscopy. Overall, 62 samples (59%) contained materials that could be diagnosed by H&E staining of filter papers fixed in formalin, and 43 samples (41%) did not contain any plaque material. Sixteen samples were diagnosed as atheromas, and 46 samples were found to contain fibrin only upon H&E staining. All 51 samples contained empty needle-shaped clefts, suggesting dissolved CCs. The median values of the long and short sides of the plaques were 42 μm (IQR 28-75μm) and 22 μm (IQR 15-47μm), respectively.

**Figure 4:** Flow chart of the detection of cholesterol crystals using direct detection and hematoxylin and eosin staining from 105 puff ruptures.

Comparison of the characteristics of plaques between puff-chandelier and puff ruptures

The ratio of visible debris from sampled puff-chandelier ruptures was higher than that from puff ruptures (26% vs. 13%; p=0.0093). The percentage of valid samples for H&E staining was higher in puff-chandelier ruptures than in puff ruptures (p=0.0009). Additionally, the detection rate of CCs was higher in puff-chandelier ruptures than that in puff ruptures (p<0.0001) and the rate of atheroma diagnosis was higher in puff-chandelier ruptures than that in puff ruptures (p<0.0095) (Table 2).

**Table 2:** Comparison of the characteristics of plaques between puff-chandelier ruptures and puff ruptures CC: cholesterol crystal

Characteristics	Puff-chandelier (N=177)	Puff (N=105)	p-value
Debris, n (%)	46 (26%)	14 (13%)	0.0093
Direct detection of CCs,			
Detection rate of CCs, n (%)	95 (54%)	21 (20%)	<0.0001
Hematoxylin and eosin staining			
Valid samples for hematoxylin and eosin staining, n (%)	135 (76%)	62 (59%)	0.0022
Detected atheromas, n (%)	51 (29%)	16 (15%)	0.0095
Detected only fibrin, n (%)	46 (26%)	36 (34%)	0.1483
The long side of plaques (μm), median (IQR)	76 (49-122)	42 (28-75)	0.0259
The short side of plaques (μm), median (IQR)	41 (24-83)	22 (15-47)	0.0286

However, there was no significant difference in the ratio of samples that contained only fibrin between the puff-chandelier and puff ruptures (p=0.1483). The ratio of undeterminable samples in puff ruptures was higher than that in puff-chandelier ruptures (p=0.0004). Furthermore, the median values of the long and short sides of the plaques in puff-chandelier ruptures were larger than those in puff ruptures (p<0.0001 and p<0.0001, respectively). The number of CCs was higher in puff chandeliers than in puff ruptures (median 0 (IQR 0-8,181)/10 mL vs. median 0 (IQR 0-0)/10 mL) (p<0.0001) (Figure 5).

**Figure 5:** Comparison of the number of CCs between puff-chandelier and puff ruptures. The number of CCs was higher in puff chandeliers than in puff ruptures (p<0.0001). CC: cholesterol crystal

The number of CCs was higher in puff-chandelier ruptures than that in puff ruptures (median 12,727 (IQR 3,636-25,909)/10 mL vs. median 3,182 (IQR 909-9,318)/10 mL in CC-positive samples (p=0.0120) (Figure 6).

**Figure 6:** Comparison of the number of CCs between puff-chandelier and puff ruptures in CC-positive samples The number of CCs was higher in puff chandeliers than in puff ruptures in CC-positive samples (p=0.0120). CC: cholesterol crystal

These results suggest that puff-chandelier ruptures tend to contain atheromas with CCs and larger plaque fragments than puff ruptures. Obtaining valid samples from puff ruptures may be more difficult because of the lower atheroma content and smaller and more easily disappearing plaque fragments than those in puff-chandelier ruptures.

IL-6 level and IL-6 ratio in puff-chandelier and puff ruptures

The IL-6 level in the sinus was 2.20 pg/mL (IQR 1.60-3.61). The IL-6 level in SRAPs was 2.75 pg/mL (IQR 2.00-6.45) for puff-chandelier ruptures and 1.75 (IQR 1.20-2.80) pg/mL for puff ruptures. There was no difference in the IL-6 levels between the puff-chandelier rupture and puff rupture (p=0.2019) (Figure 7).

**Figure 7:** Comparison between the IL-6 levels in puff-chandelier rupture and puff rupture. There was no difference in the IL-6 levels between puff-chandelier and puff ruptures (p=0.2019). IL: interleukin

The IL-6 ratio in the SRAPs was 1.15 (IQR 1.00-1.40) in puff-chandelier ruptures and 1.05 (IQR 1.00-1.17) in puff ruptures. The IL-6 ratio was higher in puff-chandelier ruptures than in puff ruptures (p=0.014) (Figure 8).

**Figure 8:** Comparison between the IL-6 ratios in puff-chandelier rupture and puff rupture. The IL-6 ratio was higher in puff-chandelier ruptures than in puff ruptures (p=0.014). IL: interleukin

The correlation between serum IL-6 levels and hs-CRP levels

There existed a moderate correlation between the levels of serum IL-6 and hs-CRP (Figure 9).

**Figure 9:** Correlation between serum IL-6 level and hs-CRP in the peripheral arteries. A significant association was observed between the levels of serum IL-6 and hs-CRP. hs-CRP: high-sensitivity C-reactive protein; IL: interleukin

A significant association was observed between the levels of serum IL-6 and hs-CRP in SRAPs (Figure 10). Variability was observed as both values increased.

**Figure 10:** Correlation between IL-6 and hs-CRP levels in spontaneously ruptured aortic plaques. A significant association was observed between the levels of serum IL-6 and hs-CRP in SRAPs. hs-CRP: high-sensitive C-reactive protein; IL: interleukin; SRAP: spontaneously ruptured aortic plaque

## Discussion

Previously, we reported the presence of various types of SRAPs [4,8] and the diversity of their constituent elements [9,13]. The contribution of SRAPs to embolism and inflammation may vary, and the degree of CCs in the SRAPs may lead to varying levels of inflammation. Following plaque rupture, free multilayered and monolayered CCs scatter from SRAPs, including puff-chandelier ruptures [3]. Macrophages recognize [18] and gather around CCs [9], triggering the production of inflammatory cytokines such as IL-1β by activating the nucleotide-binding domain, leucine-rich-containing family, pyrin domain-containing-3 (NLRP3) inflammasome in ruptured plaques [9]. IL-6 production is induced by IL-1β and IL-18 [19]. We demonstrated these processes in situ, as reported in previous studies [11,12].

Conventional analytical processes using debris sampled from catheters have a low yield rate. Only 60 (21%) of the 282 samples contained visible debris. The SRAPs have small fragments with long sides measuring <100 μm. Consequently, filter papers spread on SRAPs may contain invisible fragments. Histopathological preparation was conducted even if no apparent debris was found on the filter paper. The detection of CCs using H&E staining alone is insufficient. CCs were obtained when the surfaces of the dried filter papers appeared glittery, indicating the presence of CCs.3 When the filter paper with CCs was prepared for H&E staining, the CCs were dissolved in ethanol and xylene [1,2]. We developed a rinse method for filter paper [3,16] to improve the yield rate of direct CC detection from SRAPs and H&E staining. Direct detection methods can detect free CCs scattered by SRAPs. Direct CC detection is cheap with polarized light microscopy. The preparation did not require proficiency and took approximately five minutes after sampling. Sampling techniques, such as coronary artery sampling, can be applied to any artery [20], such as the coronary artery [21].

Puff ruptures and puff-chandelier ruptures can be distinguished by crystal glittering under fiber catheter light to estimate inflammatory levels. Plaques with abundant CCs reflect more light in NOGA than those without CCs. Puff ruptures typically contain smaller fragments and fewer CCs than puff-chandelier ruptures, and fibrin may be diminished by fibrinolysis. Thus, anticoagulant or thrombolytic therapy may be effective in treating puff ruptures. However, puff ruptures may contain few or invisible small CCs because they do not glitter under fiber catheter light, and fibrin may cause organ damage before fibrinolysis occurs.

The sampling yield rate and CC content of puff-chandelier ruptures were higher than those of puff ruptures. Additionally, puff-chandelier ruptures may cause embolisms in larger arteries and end organs because puff-chandelier segments are longer than puff ruptures. The higher IL-6 ratio in puff-chandelier ruptures indicates that the innate inflammation triggered mainly by CCs is responsible for IL-6 production [13]. Anti-inflammatory agents are expected to be more effective against puff-chandelier ruptures than puff ruptures.

Recently, inflammatory cytokine production, followed by activation of the NLRP3 inflammasome, has been identified as a target for cardiovascular diseases [9-12,16]. Colchicine is beneficial for preventing ischemic events in patients with coronary artery disease [16]. A possible mechanism for secondary prevention of cardiovascular diseases involves colchicine, which plays a vital role in reducing intracellular inflammatory responses and activating NLRP3 inflammation. This effect is mediated by the regulation of AMPK/SIRT1 signaling, leading to a decrease in cellular oxidative stress and pyroptosis in endothelial cells [22]. Patients who received an intermediate dose of canakinumab had a reduced occurrence of the primary endpoint, a composite of cardiovascular death, nonfatal acute myocardial infarction, or nonfatal stroke, accompanied by a reduction in IL-6 and CRP [14,15].

The dosage, timing, and evaluation of anti-inflammatory drug administration present challenges because of variations in the progression of atherosclerosis in the brain, heart, and aorta. Quantitative and qualitative analyses of CCs in SRAPs with NOGA sampling may serve as a precise evaluation of the overall inflammatory potential of SRAPs [10]. The inflammatory potential, such as cytokine production, of sampled SRAPs may also reveal their inflammatory potential and the effects of novel therapeutic interventions. It is essential to compare the inflammatory levels in SRAPs, indicated by biomarkers in the NLRP3 inflammasome or IL-6, with the number of CCs to assess their true reflection of the inflammatory levels in SRAPs. Moreover, the pathological manifestations of peripheral artery disease result from thrombosis, regardless of the extent of atherosclerosis [23]. There was a moderate correlation between IL-6 and hs-CRP levels throughout the body. A similar correlation was demonstrated for SRAPs. Under systemic conditions of low inflammation, IL-6 and hs-CRP levels were correlated with low viability. However, the correlation between IL-6 and hs-CRP levels was viable, especially under high inflammatory conditions.

The data on other inflammatory markers should also be examined. We plan to measure other types of interleukins, hs-CRP, and tumor necrosis factor-alpha (TNF-α) in SRAPs in future studies.

Study limitation

The assessment of SRAP inflammation levels necessitates an invasive approach. IL-6 values might be influenced by upstream blood during plaque sampling with NOGA. However, stopping blood flow for measurement is life-threatening, so this is currently the optimal method available for evaluating the inflammatory level in plaque by sampling. Training may be necessary for diagnosing CCs using polarized light microscopy [13]. Two methods for direct CC direction and H&E staining may improve CC detection, but they require more effort than conventional HE staining. 

## Conclusions

The relationship between CCs and innate inflammation in SRAPs was investigated, with a focus on variations in the CCs and IL-6 ratio in SRAPs. Plaque fragments from puff-chandelier and puff ruptures were examined, and the prevalence of CCs was found to be higher in puff-chandelier ruptures compared to puff ruptures. The number of CCs was significantly greater in puff chandeliers, indicating a potential correlation between CCs and inflammatory levels. The IL-6 ratio was also observed to be higher in puff-chandelier ruptures compared to puff ruptures.

Direct detection of CCs and H&E staining for SRAPs showed a variety of contents in terms of the degree and dimensions of CCs in puff-chandelier ruptures and puff ruptures. Puff-chandelier ruptures have more CCs that trigger innate inflammation and larger fragments than puff ruptures. NOGA can detect different characteristics and levels of inflammation as indicated by IL-6 in scattering-type SRAPs.

## References

[1] Liew YP, Bartholomew JR (2005). Atheromatous embolization. Vasc Med.

[2] Kronzon I, Saric M (2010). Cholesterol embolization syndrome. Circulation.

[3] Komatsu S, Yutani C, Ohara T, Takahashi S, Takewa M, Hirayama A, Kodama K (2018). Angioscopic evaluation of spontaneously ruptured aortic plaques. J Am Coll Cardiol.

[4] Komatsu S, Takahashi S, Yutani C, Ohara T, Takewa M, Hirayama A, Kodama K (2020). Spontaneous ruptured aortic plaque and injuries: insights for aging and acute aortic syndrome from non-obstructive general angioscopy. J Cardiol.

[5] Komatsu S, Ohara T, Takahashi S (2015). Early detection of vulnerable atherosclerotic plaque for risk reduction of acute aortic rupture and thromboemboli and atheroemboli using non-obstructive angioscopy. Circ J.

[6] Kojima K, Komatsu S, Kakuta T (2022). Aortic plaque burden predicts vascular events in patients with cardiovascular disease: the EAST-NOGA study. J Cardiol.

[7] Higuchi Y, Hirayama A, Hamanaka Y (2022). Significant contribution of aortogenic mechanism in ischemic stroke: observation of aortic plaque rupture by angioscopy. JACC Asia.

[8] Hiro T, Komatsu S, Fujii H (2018). Consensus standards for acquisition, measurement, and reporting of non-obstructive aortic angioscopy studies: a report from the Working Group of Japan Vascular Imaging Research Organization [Article in Japanese]. Angioscopy.

[9] Komatsu S, Yutani C, Takahashi S, Takewa M, Ohara T, Hirayama A, Kodama K (2022). Debris collected in-situ from spontaneously ruptured atherosclerotic plaque invariably contains large cholesterol crystals and evidence of activation of innate inflammation: Insights from non-obstructive general angioscopy. Atherosclerosis.

[10] Duewell P, Kono H, Rayner KJ (2010). NLRP3 inflammasomes are required for atherogenesis and activated by cholesterol crystals. Nature.

[11] Abela GS (2010). Cholesterol crystals piercing the arterial plaque and intima trigger local and systemic inflammation. J Clin Lipidol.

[12] Nidorf SM, Fiolet A, Abela GS (2020). Viewing atherosclerosis through a crystal lens: how the evolving structure of cholesterol crystals in atherosclerotic plaque alters its stability. J Clin Lipidol.

[13] Komatsu S, Yutani C, Takahashi S, Takewa M, Iwa N, Ohara T, Kodama K (2023). Cholesterol crystals as the main trigger of interleukin-6 production through innate inflammatory response in human spontaneously ruptured aortic plaques. J Atheroscler Thromb.

[14] Ridker PM, Everett BM, Thuren T (2017). Antiinflammatory therapy with canakinumab for atherosclerotic disease. N Engl J Med.

[15] Ridker PM, Libby P, MacFadyen JG (2018). Modulation of the interleukin-6 signalling pathway and incidence rates of atherosclerotic events and all-cause mortality: analyses from the Canakinumab Anti-Inflammatory Thrombosis Outcomes Study (CANTOS). Eur Heart J.

[16] Tardif JC, Kouz S, Waters DD (2019). Efficacy and safety of low-dose colchicine after myocardial infarction. N Engl J Med.

[17] Iwa N, Yutani C, Komatsu S, Takahashi S, Takewa M, Ohara T, Kodama K (2022). Novel methods for demonstrating human cholesterol crystals from sampled blood. Lab Med.

[18] Noda H, Yutani C, Zaima N (2022). Detection of macrophages engulfing cholesterol crystals and docosahexaenoic acid from spontaneous ruptured aortic plaque. J Cardiol Cases.

[19] Hartman J, Frishman WH (2014). Inflammation and atherosclerosis: a review of the role of interleukin-6 in the development of atherosclerosis and the potential for targeted drug therapy. Cardiol Rev.

[20] Komatsu S, Yutani C, Takewa M, Takahashi S, Kodama K (2020). Detecting free cholesterol crystals in a patient with spontaneous cholesterol embolization syndrome. JACC Case Rep.

[21] Komatsu S, Yutani C, Takahashi S, Kodama K (2020). Acute myocardial infarction caused by distal embolization from a proximal ruptured plaque. JACC Case Rep.

[22] Yang M, Lv H, Liu Q (2020). Colchicine alleviates cholesterol crystal-induced endothelial cell pyroptosis through activating AMPK/SIRT1 pathway. Oxid Med Cell Longev.

[23] Narula N, Dannenberg AJ, Olin JW (2018). Pathology of peripheral artery disease in patients with critical limb ischemia. J Am Coll Cardiol.

